RETRACTED

# Efficacy of Donepezil Hydrochloride plus Olanzapine for Senile Dementia and Its Effect on the Recovery of Cognitive Function

**DOI:** 10.1155/2022/4156312

**Published:** 2022-08-11

**Authors:** Wenxin Zheng, Xinyao Sun, Jianghua Liu

**Affiliations:** Department of Neurology, Daqing Oilfield General Hospital, Daqing, Heilongjiang, China

## Abstract

**Objective:**

To investigate the efficacy of donepezil hydrochloride plus olanzapine for senile dementia and its effect on the recovery of cognitive function.

**Methods:**

A total of 60 patients with senile dementia admitted to our hospital from April 2020 to July 2021 were recruited and assigned to receive either olanzapine alone (observation group) or donepezil hydrochloride plus olanzapine (experimental group) via the random number table method, with 30 patients in each group.

**Results:**

The combined therapy resulted in significantly higher clinical efficacy versus monotherapy of olanzapine (*P* < 0.05). Before treatment, the difference in the scores of cognitive function between the two groups did not come up to the statistical standard (*P* > 0.05). Donepezil hydrochloride plus olanzapine was associated with significantly higher scores of cognitive function in patients versus olanzapine alone (*P* < 0.05). The two groups had a similar incidence of adverse reactions (*P* > 0.05).

**Conclusion:**

Donepezil hydrochloride plus olanzapine substantially enhances the recovery of cognitive function of patients with senile dementia and features a manageable safety. Further trials are, however, required prior to clinical promotion.

## 1. Introduction

Alzheimer's disease (AD) is a common clinical neurological disease in the elder population and is characterized by mental retardation, cognitive dysfunction, and behavioral dysfunction, severely compromising quality of life [1]. Medication is the current management for senile dementia, but specific drugs have not yet been identified [2]. Hence, clinical treatment is usually performed to delay disease progression, restore cognitive function, and improve the self-care and quality of life of patients [3]. Research has reported a prevalence of AD reaching 23.3% among the elderly. AD is characterized by progressive learning and memory loss, and cognitive dysfunction, and is frequently accompanied by non-cognitive symptoms such as sleep disturbances, anxiety and fear, and activity disorders [4]. Currently, benzodiazepines are the most widely used drugs for sleep disorders, which achieve sedative-hypnotic effects through central nervous system inhibition. However, these drugs are associated with strong dependence and cognitive impairment, which restricts their application in the prevention and treatment of AD [5]. In traditional Chinese medicine (TCM), Suanzaoren Decoction is used to nourish blood and nourish yin to treat sleep disorders. Previous animal research [6] showed that Suanzaoren Decoction mediates anti-inflammatory, brain-protective, and neurotrophic effects in regulating sleep while improving spatial learning memory function in rats.

RETRACTED

Olanzapine is a common antipsychotic drug for psychiatric diseases that acts on various receptor systems and exerts various pharmacological activities [7]. Nevertheless, prior research has also reported unfavorable efficiency of olanzapine alone for senile dementia patients [8]. Donepezil hydrochloride is a common cholinesterase inhibitor that effectively inhibits the hydrolysis of acetylcholine [9] to enhance the cognitive dysfunction of patients with senile dementia. Nonetheless, it can only postpone AD progression. To this end, combined therapy of donepezil hydrochloride plus olanzapine and adjuvant TCM treatment were adopted to investigate the treatment efficiency. This study included 60 senile dementia patients treated in our hospital from April 2020 to July 2021 to evaluate the efficacy of donepezil hydrochloride plus olanzapine for senile dementia and its effect on the recovery of cognitive function.

## 2. Materials and Methods

### 2.1. Participants

A total of 60 patients with senile dementia admitted to our hospital from April 2020 to July 2021 were recruited and assigned to receive either olanzapine alone (observation group) or donepezil hydrochloride plus olanzapine (experimental group) via the random number table method, with 30 patients in each group. Undersigned informed consent was obtained from all the eligible patients, and the study protocol was approved by the hospital ethics committee, with the ethics number: SH-SY20200402. All procedures complied with the Declaration of Helsinki's ethical guidelines for clinical research.

### 2.2. Inclusion and Exclusion Criteria

Inclusion criteria were as follows: (1) patients who were clinically diagnosed with Alzheimer's disease and (2) the patients and their families were informed and voluntarily participated in this study.

Exclusion criteria were as follows: (1) patients who have recently received psychotropic drugs; (2) patients with other psychiatric diseases; and (3) patients and their families who were not willing to comply and cooperate reasonably with the present study.

### 2.3. Methods

1. The patients in the two groups received 5 mg of olanzapine (approval no. H20052688) daily at the beginning of administration, and the dose was increased according to disease severity, with a maximum of 20 mg daily [10].
2. The patients in the experimental group additionally received 5 mg of donepezil hydrochloride (H20070181) daily before bed. The dose was increased according to disease severity, with a maximum of 10 mg daily [11]. The duration of treatment was two months.

RETRACTED

*TCM Adjuvant Therapy*. The two groups received Jieyu Yizhi Decoction. The ingredients of the decoction include 12 g of Bupleuri Radix and Polygalae Radix, 30 g of Codonopsis Radix, Angelicae Sinensis Radix, Poria, Atractylodis Macrocephalae Rhizoma, and Schisandrae Chinensis Fructus, 9 g of Pinelliae Rhizoma, 15 g of Paeoniae Radix Alba and Acori Tatarinowii Rhizoma, and 10 g of Licorice. The herbs were decocted with water to obtain 200 mL of filtrate and administered twice daily. Benzodiazepines were prevented during TCM treatment.

### 2.4. Outcome Measures

#### 2.4.1. Clinical Efficacy

  Cured: the patient's BEHAVE-AD score decreased by less than 75% after treatment.
  Markedly effective: the patient's BEHAVE-AD score decreased by 50–75% after treatment.
  Effective: the patient's BEHAVE-AD score after treatment decreased by 25–50%.
  Ineffective: the patient's BEHAVE-AD score after treatment decreased by less than 25%.

#### 2.4.2. Cognitive Function Score

Wechsler Adult Intelligence Test and Clinical Memory Scale were used to evaluate the cognitive function of patients, including image-free recall, recognition of meaningless images, pointing memory, memory of portrait characteristics, learning association, memory IQ, speech IQ, operational IQ, and total IQ. The higher the score of each index, the better the recovery of the cognitive function of the patient.

#### 2.4.3. Adverse Reactions

Adverse reactions during treatment include insomnia, lethargy, nausea and vomiting, and abnormal liver function.

### 2.5. Statistical Analysis

SPSS 21.0 was the software used for data analyses. Measurement data were expressed as $\left(\bar{x}\pm s\right)$ and analyzed using the independent sample *T* test. Count data were expressed as the number of cases (rate) and analyzed using the chi-square test. Statistical significance was indicated by *P* < 0.05.

## 3. Results

### 3.1. Patient Characteristics

There were 19 males and 11 females in the observation group, aged 62 to 81 (73.27 ± 3.35) years, with disease duration of 1 to 7 (3.82 ± 0.58) years. There were 22 males and 8 females in the experimental group, aged 61 to 83 (73.44 ± 3.42) years. The patient characteristics of the two groups were comparable (*P* > 0.05) (Table 1).

### 3.2. Comparison of Clinical Efficacy

The combined therapy resulted in significantly higher clinical efficacy versus monotherapy of olanzapine (*P* < 0.05) (Table 2).

RETRACTED

### 3.3. Cognitive Function Score Comparison

Before treatment, the difference in the scores of cognitive function between the two groups did not come up to the statistical standard (*P* > 0.05). Donepezil hydrochloride plus olanzapine was associated with significantly higher scores of cognitive function in patients versus olanzapine alone (*P* < 0.05) (Table 3).

### 3.4. Comparison of Adverse Reactions

There was no statistically significant difference in the incidence of adverse events between the two groups (*P* > 0.05) (Table 4).

## 4. Discussion

Senile dementia, also known as Alzheimer's disease, is a common central nervous system degenerative disease in the elderly [12]. It is associated with severe cognitive and behavioral disorders and even mental disorders. Research has revealed that the leading causes of Alzheimer's disease are amyloid deposition, neurofibrillary tangles, and decreased levels of acetylcholine in the brain's neurotransmitters, resulting in a continuous decrease in the number of neurons and compromised memory [13]. Symptoms of dementia patients include delusions and agitation. At present, antipsychotic drugs are mainly used for the clinical management of senile dementia, but specific drugs for the disease are still unavailable [14]. At present, the western drug treatment for Alzheimer's disease mainly includes [15] (i) choline acetyltransferase (AChE) inhibitors; (ii) antipsychotic drugs and anti-anxiety and depression drugs (risperidone, fluoxetine, and buspirone); and (iii) neuroprotective agents. However, these drugs only temporarily alleviate cognitive impairment and its associated abnormal behaviors and are associated with poor patient intolerance and compliance and a cascade of adverse events such as nausea and vomiting, dizziness, diarrhea, and delayed-onset dyskinesia. Alzheimer's disease belongs to the category of dementia in TCM [16], and the onset of this disease is related to three key factors: deficiency, phlegm, and stasis, so its management mostly involves tonifying the kidney and strengthening the spleen, dispelling phlegm, and activating blood circulation to resolve stasis.

Olanzapine is a new clinical atypical neuroleptic drug [17] with a strong affinity with serotonin, dopamine D, and histamine receptors. It effectively blocks D2 and HT2A receptors. The secretion of dopamine significantly relieves patients' mental symptoms such as delusions, hallucinations, and destructive emotions [18]. Donepezil hydrochloride, as a common clinical cholinesterase inhibitor, effectively inhibits the hydrolysis of acetylcholine by acetylcholinesterase and increases the level of acetylcholine in the synaptic space, thus enhancing the role of acetylcholine in the central nervous system [19]. Devanand et al. [20] indicated that donepezil hydrochloride could effectively improve the dementia behavior and cognitive function of patients with Alzheimer's disease. Eskandary et al. [21] have shown that the single use of donepezil hydrochloride or olanzapine in patients with Alzheimer's disease is suboptimal. Matsunaga et al. [22] also showed that joint administration of drugs could effectively relieve the symptoms of Alzheimer's disease.

RETRACTED

The results of the present study showed that the donepezil hydrochloride plus olanzapine was associated with significantly higher clinical efficacy and scores of cognitive function in patients versus olanzapine alone (*P* < 0.05), indicating a favorable treatment efficiency of donepezil hydrochloride plus olanzapine for senile dementia. It effectively increases the concentration of acetylcholine in the relevant areas of the patient's brain, which positively affects the cognitive status of the patient's body function [23]. The reason may be that donepezil hydrochloride regulates the hydrolysis of acetylcholine ester in the central neurons, boosts the level of acetylcholine in brain tissue, and alleviates memory loss and mental agitation in Alzheimer's disease patients [24]. Moreover, the patients in the present study received TCM adjuvant therapy. In the Jieyu Yizhi Decoction, Bupleuri Radix detoxifies the liver and regulates liver qi, Codonopsis Radix and Angelicae Sinensis Radix, as the monarch drug, strengthen the spleen, benefit the qi, and tonify the blood, Poria and Atractylodis Macrocephalae Rhizoma strengthen the spleen and resolve dampness, Schisandrae Chinensis Fructus nourishes blood and softens liver, Pinelliae Rhizoma dries dampness and resolves phlegm, Paeoniae Radix Alba and Polygalae Radix clear phlegm and invigorate the brain, Acori Tatarinowii Rhizoma tonifies the kidneys, and Licorice harmonizes all the medicines. Curcumae Radix, Cyperi Rhizoma, and Chuanxiong Rhizoma can be added for elderly female patients to enhance the liver detoxification, and Epimedii Folium, Eucommiae Cortex, and Taxilli Herba can be added for elderly male patients to tonify the kidney. The dosages of Acori Tatarinowii Rhizoma and Polygalae Radix can be increased in obese patients, and Crataegi Fructus and lotus leaves can be added. If the disease has been prolonged and there are signs of blood stasis, Tongqiao Huoxue Decoction was administered.

Donepezil hydrochloride plus olanzapine herein significantly improved the cognitive function of patients and considerably relieved the disease condition of patients with Alzheimer's disease [25]. There was no statistically significant difference in the incidence of adverse reactions between the two groups of patients, which indicated a manageable safety of the combined therapy of donepezil hydrochloride plus olanzapine [26, 27].

RETRACTED

In conclusion, donepezil hydrochloride plus olanzapine substantially enhances the recovery of cognitive function of patients with senile dementia and features a manageable safety. Further trials are, however, required prior to clinical promotion.

## Figures and Tables

**Table 1:** Patient characteristics $\left(\bar{x}\pm s,n\left(\%\right)\right)$.

	Observation group (*n*=30)	Experimental group (*n*=30)	t (*t*/*x*^2^)	*P* value
Gender			0.693	0.405
Male	19	22		
Female	11	8		

Age (years)	62 − 81	61 − 83		
Average age (years)	73.27 ± 3.35	73.44 ± 3.42	−0.194	0.847
Disease duration (years)	1 − 7	1 − 8		
Average disease duration (years)	3.82 ± 0.58	3.94 ± 0.61	−0.781	0.438

**Table 2:** Comparison of clinical efficacy (*n*(%)).

Group	*n*	Cured	Markedly effective	Effective	In effective	Total efficiency (%)
Observation group	30	6	10	6	8	22 (73%)
Experimental group	30	10	8	11	1	29 (97%)
*x* ^2^	—		—	—	—	6.405
*P*	—		—	—	—	0.011

**Table 3:** Cognitive function score comparison $\left(\bar{x}\pm s\right)$.

Indices	Time	Observation group (*n*=30)	Experimental group (*n*=30)	*t*	*P*
Image-free recall	Before therapy	12.67 ± 2.43	12.68 ± 2.43	−0.016	0.987
	After treatment	13.66 ± 2.79	17.87 ± 3.13	−5.499	<0.001

Recognition of meaningless images	Before therapy	15.46 ± 3.11	15.42 ± 3.09	0.05	0.96
	After treatment	16.64 ± 2.80	19.70 ± 3.25	−3.907	<0.001

Pointing memory	Before therapy	9.53 ± 1.25	9.45 ± 1.48	0.226	0.822
	After treatment	10.72 ± 1.84	13.78 ± 2.36	−5.601	<0.001

Portrait feature memory	Before therapy	12.45 ± 2.18	12.35 ± 2.43	0.168	0.867
	After treatment	13.06 ± 1.83	15.71 ± 2.25	−5.005	<0.001

Learning association	Before therapy	11.49 ± 2.32	11.43 ± 2.31	0.1	0.921
	After treatment	12.05 ± 2.47	16.09 ± 2.66	−6.096	<0.001

Memory IQ	Before therapy	77.45 ± 5.53	77.54 ± 5.48	−0.063	0.95
	After treatment	83.69 ± 5.66	90.65 ± 6.19	−4.545	<0.001

Speech IQ	Before therapy	82.42 ± 3.85	83.41 ± 4.15	−0.958	0.342
	After treatment	85.86 ± 4.53	91.78 ± 5.26	−4.671	<0.001

Operational IQ	Before therapy	77.05 ± 4.28	76.95 ± 4.35	0.09	0.929
	After treatment	79.78 ± 4.30	83.68 ± 4.28	−3.521	<0.001

Total IQ	Before therapy	82.59 ± 4.52	82.63 ± 4.35	−0.035	0.972
	After treatment	85.76 ± 4.69	90.81 ± 5.15	−3.971	<0.001

**Table 4:** Comparison of adverse reactions (*n* (%)).

	Observation group (*n* = 30)	Experimental group (*n* = 30)	x^2^	*P* value
Insomnia	1	2		
Lethargy	1	1		
Feeling sick and vomiting	1	1		
Abnormal liver function	0	0		
Overall incidence (%)	3 (10%)	4 (13%)	0.162	0.688

RETRACTED

## Data Availability

No data were used to support this study.
